# Clinical Orodental Anomalies in Taiwanese Children under Age Six: a Study Based on the 1995-1997 National Dental Survey

**DOI:** 10.1155/2020/2056340

**Published:** 2020-07-19

**Authors:** Po-Sen Chang, Tzung-Hai Yen, Chun-Jui Huang, Amy Ming-Fang Yen, Sam Li-Sheng Chen, Aileen I. Tsai

**Affiliations:** ^1^Department of Pediatric Dentistry, Chang Gung Memorial Hospital, Linkou, Taiwan; ^2^Department of Nephrology and Clinical Poison Center, Chang Gung Memorial Hospital and College of Medicine, Chang Gung University, Linkou, Taiwan; ^3^Kidney Research Center, Chang Gung Memorial Hospital, Linkou, Taiwan; ^4^Center for Tissue Engineering, Chang Gung Memorial Hospital, Linkou, Taiwan; ^5^Division of Endocrinology and Metabolism, Department of Medicine, Taipei Veterans General Hospital, Taipei, Taiwan; ^6^Faculty of Medicine, School of Medicine, National Yang-Ming University, Taipei, Taiwan; ^7^School of Oral Hygiene, College of Oral Medicine, Taipei Medical University, Taipei, Taiwan

## Abstract

There are few published studies that report the prevalence of intraoral anomalies for young children. The purpose of this study was to investigate the prevalence and distribution of several congenital oral and paraoral anomalies in Taiwanese children under age six. Twenty-five cities and townships were randomly sampled in different areas of Taiwan using the stratified method. These cities and townships represent cross-sectional samples of geographic locations and socioeconomic levels. A total of 981 Taiwanese children under age six were examined with dental mirrors and explorers as part of the national dental survey. The results of this survey indicated an 11.31% prevalence of geographic tongue. This number is higher than that reported in studies previously performed in different countries. The occurrence of double teeth in primary dentition was found to be 2.14%. Ankyloglossia had a frequency of 1.22%, and primary talon cusp a frequency of 0.61%. Seven (0.71%) children exhibited fissured tongues. Thirteen (1.33%) cases of hypodontia were found. These values were different from those reported in several other countries, which may be attributed to differences in the ethnic and racial composition of the population studied.

## 1. Introduction

The presence of orodental anomalies is relatively common during routine oral examination. Many epidemiological studies in several countries have reported prevalence values for various orodental anomalies, such as those affecting the tongue, frenum, gingiva, number of teeth, shape of teeth, size of teeth, and even color of teeth [1–89]. Epidemiological studies of orodental anomalies are still lacking in published reports compared with reports regarding dental caries, periodontal diseases, and oral cancer. Dental anomalies of number, shape, and size may occur in primary and permanent dentitions. Most of these reports are representative of oral and paraoral lesions in either adult or schoolchildren populations [18, 20, 21, 28–30]. There have been few publications regarding the occurrence and frequency of certain orodental anomalies in young children.

In addition, most of the studies have focused on non-Asian races [1–6, 8–10, 12, 13, 15–22, 24, 25, 27–35, 37–41, 43, 46, 48, 51, 52, 54–61, 63–69, 71, 73–76, 78–80, 86–89], and many orodental anomalies often have a considerable relationship with race. In understanding the prevalence of orodental anomalies in children in Taiwan, national dental surveys can be studied as a reference for public health planning and activities [13, 33, 59] and as a basis for prevention policies. Huang et al. demonstrated the prevalence of mesiodens in Taiwanese children aged 2.5 and 7 years in a hospital [36]. Liu and Huang investigated the prevalence of oral abnormalities such as palatal cysts and gingival cysts in Taiwanese newborns in a hospital [56]. Chen et al. reported the prevalence of dental anomalies such as hypodontia, hyperdontia, and double teeth in Taiwanese preschool children [72]. As mentioned by Wu et al., the prevalence of double primary teeth in the dental records of Taiwanese children under 17 years old is 0.72% [73].

Selecting a representative sample of infants and toddlers is usually difficult because these children are not readily accessible [90, 91]. Thus, there is a paucity of dental health data from birth to 6 years of age in the Taiwanese population [56, 72] as well as worldwide. The first national dental survey of children younger than the age of 6 in Taiwan, conducted from 1995 to 1997, provides useful orodental health epidemiological data, including caries status and orodental anomalies. Although the execution of this nationwide study was in 1995 to 1997, the prevalence of orodental anomalies usually represents a genetic and racial composition and has a rather stable range of values.

The purpose of this study was to investigate the prevalence and distribution of several congenital oral and paraoral anomalies in Taiwanese children under age six in a nationwide dental survey.

## 2. Materials and Methods

This cross-sectional descriptive study was conducted from 1995 to 1997. The investigation was approved by the Institutional Review Board of Chang Gung Memorial Hospital (IRB number: 201600095B0C502) and followed the methods described in our previous study [92], including the following:

### 2.1. Sample Design

There are 309 cities, villages, and townships in Taiwan, according to the Republic of China's Ministry of the Interior. These geographic locations are divided into 10 administrative strata as follows: (1) developing area, (2) mountainous area, (3) industrial area, (4) hilly area, (5) remote area, (6) service business area, (7) combination area, (8) metropolitan area in Taipei City (northern area of Taiwan), (9) metropolitan area in Kaohsiung City (southern area of Taiwan), and (10) five well-developed county administration centers according to their socioeconomic status (SES) and degree of urbanization.

The sample design in this study was based on the principle of stratification, using multistage sampling with unequal sample probability. We designated the population elements into these 10 strata. All characteristics, such as location, age, and sex, and each population group appeared in our sample. The population of interest in this investigation was Taiwanese children under age 6; children in orphanages were excluded.

### 2.2. Multistage Sampling

Two-stage sampling was conducted within each stratum to assure random sampling in this survey. In the first stage, the probabilities proportional to sizes (PPS) method was conducted to select districts from 10 strata. In addition, the number of sampling districts for each stratum was proportional to the number of children under age 6 within each stratum. There were 25 districts selected in this study. The second stage was the selection of 15 blocks from each sampled district using cluster sampling. There were 15 geographical neighbor house units within each block. Therefore, each sampled district was composed of 225 (15x15) household samples. In each house sample, children under age 6 were the subjects of this survey.

### 2.3. Selection of Blocks

The position of each district on the map utilized computer-selected two-dimensional random coordinate points. A valid coordinate point determined the first house unit of a sampling block and contained 15 neighboring house units within a radius of 100 meters.

Maps were a major factor in our survey. However, the most recent and precise distribution of all streets could not be completely depicted by current maps. Hence, in the process of selecting blocks, the position of the first house units was determined by a global positioning system (GPS).

### 2.4. Selection of House Units and Sampling Objects

Fifteen sampling house units for each sampled block had to be neighbors with each other geographically. That is, sampling house units for each block could not be separated by rivers or main avenues. In addition, companies, schools, and dormitories were excluded from sampling house units.

All children under age 6 living in sampling houses were regarded as sampling objects. Children who were absent from the household during the survey were asked to take the examination on the following day. If the child was not available on the following day, he/she was excluded from the study.

### 2.5. Order of Interviews

To avoid a seasonal influence on the rate of children available for oral/dental examination, we randomly selected the order of interviews for 25 sampled districts. In addition, visitors were sent to each house in random the sample to introduce the survey and to invite the family to participate in this survey. All eligible people in the house units were interviewed, and a specially designed survey questionnaire was used. If there were children under the age of 6 in the house unit, the child would be scheduled for an oral/dental examination.

A total of 5625 house units were sampled, and 1681 house units had children under the age of 6. A total of 981 children were available for oral/dental examinations using dental mirrors, explorers, disposable tongue depressors, and natural and/or artificial light. Specially designed charts were used to record personal data and oral conditions. Dental radiographs were not taken. The oral/dental examinations were performed by 3 pediatric dentists. Before the survey, the diagnostic criteria and calibration were thoroughly discussed. The examination procedure, instruments used, and diagnostic criteria were based on WHO guidelines [93].

Parental interviews were carried out by trained interviewers. The parent or the caregiver was also asked to complete a questionnaire about their child that provided demographic information, such as the child's age and sex.

Interexaminer calibration was performed by comparing independent oral/dental examinations of randomly selected children. Calibration studies were carried out in a local kindergarten in which twenty 3- to 5-year-old children were assessed. Values for kappa statistics for the interexaminer agreement were 0.97 and 0.98. These values included caries status and all oral conditions diagnosed.

### 2.6. Diagnostic Criteria

The following criteria for a positive finding were used to diagnose the selected conditions being investigated.

#### 2.6.1. Tongue

1. Ankyloglossia (tongue tie) is a thick frenum on the ventral surface of the tongue that does not allow protrusion of the tip of the tongue beyond the vermilion border of the lower lip.
2. Fissured tongues are multiple linear fissures of various depths on the dorsal surface of the tongue.
3. Geographic tongue (benign migratory glossitis) is a patchy area of papillary atrophy with partly sharp demarcations partially surrounded by white lines.
4. Median rhomboid glossitis is a red zone that varies in size with no filiform papillae. This is located on the midline and anterior to the posterior third of the dorsum of the tongue.

#### 2.6.2. Oral Mucosa

1. Fordyce granules are single or multiple, yellow papules that vary in size, found in the buccal mucosa, unilaterally or bilaterally, and/or the vermilion border of the lip.
2. Gingival cysts are small, elevated, yellow to pink multiple nodules in the neonatal palate and alveolar ridges.

#### 2.6.3. Palate

1. Torus palatinus is a bony convexity on the palatal surface of the maxilla.

#### 2.6.4. Mandible

1. Torus mandibularis is a bony convexity on the lingual surface of the body of the mandible.

#### 2.6.5. Teeth

1. Double teeth are any two teeth partially or completely joined at their crowns or a total or partial division of the crown of a single tooth. No clinical distinction was made between fusion and gemination.
2. Hyperdontia is the number of teeth that exceeds the normal amount in either primary or permanent dentition.
3. Hypodontia is a congenital absence of one or more primary or permanent teeth.
4. Natal teeth are defined as the presence of teeth at birth.
5. Neonatal teeth appear between the first and thirtieth day of life.
6. Peg lateral incisors are maxillary or mandibular lateral incisors that are conical in shape, lacking the normal parallel or flared mesial and distal surfaces.
7. Talon cusp is a form of supernumerary cusp seen on the cingulum portion of the tooth usually extending and protruding to the incisal edges.

### 2.7. Statistics

The data collected were processed and analyzed using SPSS statistics version 19.0 software (SPSS, Chicago, IL, USA). The chi-square test was used to analyze the association between orodental anomalies and sex. *P* < 0.05 was considered statistically significant.

## 3. Results

The randomly selected sample of children in this study provided an estimate of the oral condition of the 1.9 million children between the ages of 0 and 6 years in Taiwan.

In this study, 5625 house units were sampled. A total of 1681 house units had children under 6. A total of 981 children were available for oral/dental examination; 526 (53.62%) were boys, and 455 (46.38%) were girls. The sex ratio of 1.16 boys per girl is within the accepted range. The distribution of the age groups of the 981 children is presented in Table 1.

Table 2 shows the orodental anomalies of 981 young children. All the selected entities of anomalies, except hypodontia, appeared to affect both males and females comparably. Hypodontia appeared to be more common in females than in males (*P* = 0.026).

Table 3 shows the cases with double teeth, hyperdontia, hypodontia, and talon cusp. Seven of the 22 double teeth cases occurred between the mandibular right cuspid and lateral incisor. The second most frequent incidence of double teeth occurred at the mandibular left central and lateral incisor. Three out of 9 talon cusps occurred on the left maxillary central incisors.

There was only one child who had a supernumerary tooth and it was visible without radiography. The most common congenitally absent primary tooth was the right mandibular lateral incisor.

None of the following anomalies or conditions was found: median rhomboid glossitis, Fordyce granules, torus palatinus, or torus mandibularis. There was one child who was reported to have a natal tooth. However, that natal tooth was not seen at the time of this study.

The prevalence values of orodental anomalies in young children from various published sources are summarized in Table 4. The previously reported numbers were also compared with those of the present study for the conditions studied.

## 4. Discussion

This is the first national survey of orodental anomalies of Taiwanese children under age 6. The data were derived from a nationwide investigation of oral health from 1995 to 1997. The data used for analysis were derived from our previous caries investigation study [92]. The estimated caries prevalence ranged from 5% to 89% across different age groups based on 981 children. The 981 samples might be sufficient for caries investigation according to the calculated sample recommendation from a prevalence study by Pourhoseingholi et al. [94]. The sample size was 1825 if the prevalence was as low as 5%. Thus, we might need more samples for some rare disease investigations in the current study. Although our samples are quite consistent with the population distribution indicated in the 1995 national census, the estimated prevalence for some diseases due to an insufficient sample size might suggest bias, creating a limitation. Therefore, a more current survey should be conducted for more updated information.

### 4.1. Fissured Tongue

In the present study, we found 7 children (0.71%) with this condition. Chosack et al. and Halperin and coworkers reported a steady rise in the prevalence of fissured tongue that increases with age [5, 21]. Our number is lower than those previously reported [28, 31, 33, 54], which can possibly be attributed to age and ethnic factors.

### 4.2. Geographic Tongue

Prevalence reports for this condition have varied in the literature from 0.16% to 14.29%, depending on the population studied. Redman stated that geographic tongue was more common in females [18]. Prinz reported a 5 : 3 female to male ratio [1]; however, neither the number of subjects involved nor the method of selection was explained. Our observations found this condition to be equally frequent in both sexes, with overall prevalence values of 11%. The findings of Turpin and Caratzali suggest that geographic tongue is more common in children [2]. Mani also reported that geographic tongue maintained a lower prevalence rate in older age groups [32]. Redman suggested that the peak age for this condition was 2 to 3 years of age [18]. This may explain the higher prevalence value of this condition in our study because the population studied was children aged 0 to 6 years. Togo reported very high rates of occurrence of this condition among Japanese children (up to 8%) [12]. Rahamimoff and Muhsam studied Israeli children and reported a rate of 14% [9]. Thus, these high rates suggest that this condition may be due to ethnic factors.

There was one observation of a child with a combination of both fissured tongue and geographic tongue.

### 4.3. Gingival Cyst

Two infants, a one-month-old boy and a 10-month-old girl, were identified. Usually, cysts are transient and degenerate early in infancy. In this survey, there were 114 children under age one. Therefore, gingival cysts were represented in 2 out of 114 infants (1.75%).

This study included a population of children aged 0-6 years. Some of them did not have any teeth. The abnormalities of their dentition are discussed below.

### 4.4. Double Teeth

Double teeth were seen in nine (1.71%) boys and twelve (2.64%) girls, with an average of 2.14% for both sexes combined. The sex difference was statistically insignificant. Our findings show a higher prevalence for double teeth than those in previous reports [8, 13, 19, 24, 30, 35, 41]. Ethnic and genetic composition may account for this disparity. Clayton stated that fused teeth were more commonly found in the 3-5 year age group and were equally distributed between males and females [8]. However, Sedano et al. and Buenviaje and Rapp reported that fused teeth were more common among males [29, 33]. This study and previous reports in the literature [8, 13, 30] indicate that double teeth were usually observed in the incisor-canine area of either jaw.

### 4.5. Hypodontia

The frequency of hypodontia in our study was 1.33%. The present study shows a higher prevalence with greater predilection towards females (*P* = 0.026). Most of the missing teeth involved lateral incisors [8, 19, 25, 42, 72]. Our study confirms that the teeth most commonly missing were mandibular lateral incisors [42, 72].

### 4.6. Hyperdontia and Peg Lateral Incisor

In the present study, both conditions had low prevalence values. However, since dental radiographs of this population were not taken, some unerupted supernumerary teeth may have remained undiscovered. Two peg lateral incisors occurred on the mandible. Our 0.2% prevalence for primary peg lateral incisors is similar to the frequency reported by Clayton [8].

### 4.7. Talon Cusp

Talon cusp has been reported in both permanent and primary dentitions [39]. This anomaly occurred three times more often in permanent dentition than in primary dentition [39]. To date, more than 100 cases of talon cusps on the primary incisors of normal children have been reported in the literature [58, 61, 63–66, 71, 75, 76, 78, 80]. Our present study found 6 children (3 boys and 3 girls) with a total of 9 talon cusps.

The developmental anomalies of primary teeth may affect esthetic and dental caries along the fusion fissures, periodontal problems, delayed or ectopic eruption of the permanent successors, and orthodontic problems. Early detection of these orodental anomalies contributes to dental treatment planning and precludes any of the adverse effects of these abnormalities on permanent dentition.

The data derived from the nationwide survey can be used not only in clinical dental practice but also in future anthropologic or genetic research.

## 5. Conclusions

In conclusion, the most common orodental anomaly among young children in Taiwan in this survey was geographic tongue (11.31%). The next most common anomalies and rates were double teeth, 2.07%, and hypodontia, 1.28%. These data provide a useful reference for the prevalence of orodental anomalies and can be used as a basis for public health planning activities.

## Figures and Tables

**Table 1:** The distribution of young children in Taiwan according to age.

	Age (year)					
	0-1	1-2	2-3	3-4	4-5	5-6
No.	114	182	182	178	147	178
Percent	11.62	18.55	18.55	18.14	14.98	18.14

**Table 2:** The distribution of orodental anomalies according to sex in young children in Taiwan.

Orodental anomalies	Male (*n* = 526, 53.62%)		Female (*n* = 455, 46.38%)		Total (*n* = 981)		*P* value
	*n*	%	*n*	%	*n*	%	
Ankyloglossia	7	1.33	5	1.10	12	1.22	0.742
Fissured tongue	5	0.95	2	0.44	7	0.71	0.343
Geographic tongue	59	11.22	52	11.43	111	11.31	0.917
Gingival cyst	1	0.19	1	0.22	2	0.20	0.918
Double teeth	9	1.71	12	2.64	21	2.14	0.317
Hyperdontia	1	0.19	0	0	1	0.10	0.352
Hypodontia	3	0.57	10	2.20	13	1.33	0.026^∗^
Peg lateral incisor	1	0.19	1	0.22	2	0.20	0.918
Talon cusp	3	0.57	3	0.66	6	0.61	0.858

^∗^Statistically significant, according to sex (*P* < 0.05).

**Table 3:** The distribution of teeth affected by double teeth, hyperdontia, hypodontia, and talon cusp.

Double teeth		Hyperdontia		Hypodontia		Talon cusp	
Tooth	No. of teeth affected	Tooth	No. of teeth affected	Tooth	No. of teeth affected	Tooth	No. of teeth affected
61-62	3	72	1	52	3	51	2
71-72	5			62	2	53	1
72-73	4			72	2	61	3
81-82	3			73	4	62	1
82-83	7			82	5	63	2
				83	4		
Total	22		1		20		9

**Table:** (a) Previous prevalence studies of orodental anomalies in young children

First author	Country	Sample size	Age group	Ankyloglossia	Fissured tongue	Geographic tongue	Gingival cyst
Rahamimoff, 1957 [9]	Israel	5425	0-2	—	—	14.29	—
Moller, 1963 [13]	Iceland	609	2-7	—	—	0.16	—
Ghose, 1982 [26]	Iraq	859	6	—	0.93	3.61	—
Jorgenson, 1982 [27]	USA	2164	Neonate	1.80	—	—	43.72
Friend, 1990 [34]	USA	500	Neonate	4.4	—	—	25.0
Flinck, 1994 [38]	Sweden	1021	Neonate	2.45	—	—	21.94
Bezerra, 2000 [45]	Brazil	1042	0-5	—	—	0.48	0.86
Messner, 2000 [46]	USA	1041	Neonate	4.8	—	—	—
Baldani, 2001 [49]	Brazil	200	0-2	—	—	5.0	—
Ballard, 2002 [51]	USA	3036	Neonate	4.18	—	—	—
Vörös-Balog, 2003 [54]	Hungary	159	1-5	—	18.23	6.92	—
Bessa, 2004 [55]	Brazil	746	0-4	0.67	0.54	9.92	1.34
Liu, 2004 [56]	Taiwan	420	Neonate	—	—	—	79
Hogan, 2005 [57]	UK	1866	Neonate	10.77	—	—	—
Ricke, 2005 [60]	USA	3490	Neonate	4.24	—	—	—
Paula, 2006 [62]	Brazil	561	Neonate	—	—	—	28.16
Freudenberger, 2008 [67]	Mexico	2182	Neonate	10.6	—	—	96.9
George, 2008 [68]	India	1038	Neonate	—	—	—	13.78
Çetinkaya, 2011 [74]	Turkey	2021	Neonate	0.3	—	—	15.19
Monteagudo, 2012 [79]	Spain	1000	Neonate	—	—	—	13.4
Vieira-Andrade, 2013 [81]	Brazil	541	0-5	—	0.55	2.77	—
Kumar, 2017 [85]	India	25786	Neonate	0.52	—	—	—
Perez-Aguirre, 2018 [87]	Mexico	2216	Neonate	1.49	—	—	79
de Oliverira, 2019 [88]	Brazil	400	Neonate	9.0	—	—	23.0
Present study	Taiwan	981	0-6	1.22	0.71	11.31	0.20

**Table:** (b) Previous prevalence studies of orodental anomalies in young children (continued)

First author	Country	Sample size	Age group	Double teeth	Hyperdontia	Hypodontia	Peg lateral incisor	Talon cusp
Plaetschke, 1938 [3]	Poland	1000	^∗^	0.5	0.2	0.7	—	—
Tinn, 1940 [4]	UK	8500	^∗^	0.3	—	—	—	—
Leighton, 1953 [6]	UK	2700	^∗^	—	0.8	0.9	—	—
Menczer, 1955 [7]	USA	2209	^∗^	0.14	0.25	0.1	—	—
Clayton, 1956 [8]	USA	1795	3-5	0.8	1.8	4.6	—	—
Saito, 1959 [10]	Japan	7589	^∗^	4.5	—	0.2	—	—
Grahnén, 1961 [11]	Sweden	1173	^∗^	0.5	0.3	0.4	—	—
Moller, 1963 [13]	Iceland	609	2-7	0.16	0.82	0.16	—	—
Niswander, 1963 [14]	Japan	285	^∗^	2.46	—	—	—	—
Turobova, 1965 [15]	USSR	3520	^∗^	0.7	—	—	—	—
Curzon, 1967 [16]	Canada	776	^∗^	0.9	0.6	0	—	—
Toth, 1967 [17]	Germany	2539	^∗^	0.6	—	—	—	—
Ravn, 1971 [19]	Denmark	4564	3	0.85	0.55	0.55	—	—
Brook, 1974 [20]	UK	741	^∗^	1.6	0.8	0.3	—	—
Holm, 1974 [22]	Sweden	208	3	0.5	1.4	0.5	—	—
Rasmussen, 1975 [23]	Denmark	406	^∗^	—	1.7	0.2	—	—
Järvinen, 1980 [24]	Finland	1141	3-4	0.70	—	—	—	—
Järvinen, 1981 [25]	Finland	1141	3-4	—	0.44	0.88	—	—
Magnússon, 1984 [30]	Iceland	572	0-7	0.70	0.5	0.5	—	—
Skrinjarić, 1991 [35]	Croatia	2987	3-6	0.43	0.10	0.47	—	—
Jones, 1993 [37]	USA	493	3-4	0.41	0.20	0	—	—
Ooshima, 1996 [40]	Japan	905	3-6	—	—	—	1.2	0.6
Whittington, 1996 [41]	New Zealand	1680	5	0.83	0.18	0.35	—	—
Yonezu, 1997 [42]	Japan	2733	3	4.10	0.07	2.38	0.55	—
Carvalho, 1998 [43]	Belgium	750	3-5	0.67	0.80	0.42	—	—
Aguiló, 1999 [44]	Spain	6000	^∗^	0.8	—	—	—	—
Miyoshi, 2000 [47]	Japan	8122	3-6	—	0.05	—	—	—
Bäckman, 2001 [48]	Sweden	739	7	—	—	—	0.8	—
Tasa, 2001 [50]	India	412	6	1.46	—	—	—	—
Cheng, 2003 [53]	China	4286	2-6	1.52	—	—	—	—
King, 2008 [69]	Hong Kong, China	936	5	4.06	2.78	4.06	—	0.53
Kramer, 2008 [70]	Brazil	1260	2-5	1.27	0.32	0.63	—	—
Chen, 2010 [72]	Taiwan	2611	2-6	2.91	0.27	1.80	—	—
Kapdan, 2012 [77]	Turkey	1149	2-5	1.31	0.26	0.17	—	—
Mukhopadhyay, 2014 [82]	Bangladesh	2757	4-6	0.40	0.40	0.51	—	0.07
Deolia, 2015 [83]	India	1398	2-5	2.36	0.36	0.64	—	—
Lochib, 2015 [84]	India	1000	3-5	0.5	—	0.4	—	—
Shilpa, 2017 [86]	India	4180	3.5-6	0.95	0.21	0.88	—	0.04
Folayan, 2019 [89]	Nigeria	918	3-5	0.44	1.20	0.87	1.20	0.65
Present study	Taiwan	981	0-6	2.14	0.10	1.33	0.20	0.61

^∗^Primary dentition.

## Data Availability

The data used to support the findings of this study are available from the corresponding author upon request.
